This article has been retracted.

# Contact/Release Coordinated Antibacterial Cotton Fabrics Coated with N-Halamine and Cationic Antibacterial Agent for Durable Bacteria-Killing Application

**DOI:** 10.3390/ijms21186531

**Published:** 2020-09-07

**Authors:** Hua Han, Chang Liu, Jie Zhu, Fa-Xue Li, Xue-Li Wang, Jian-Yong Yu, Xiao-Hong Qin, De-Qun Wu

**Affiliations:** 1 Key Laboratory of Textile Science & Technology, Ministry Education, College of Textiles, Donghua University, No.2999 North Renmin Road, Songjiang, Shanghai 201620, China; 1159120@mail.dhu.edu.cn (H.H.); 2180068@mail.dhu.edu.cn (C.L.); fxlee@dhu.edu.cn (F.-X.L.); wxl@dhu.edu.cn (X.-L.W.); yujy@dhu.edu.cn (J.-Y.Y.); 2 School of Textiles and Fashion, Shanghai University of Engineering Science, No.333 Longteng Road, Songjiang, Shanghai 201620, China; 09190006@sues.edu.cn; 3 Innovation Center for Textile Science and Technology, Donghua University, Shanghai 201620, China

**Keywords:** antibacterial, durable, cotton fabrics, chemical modification

## Abstract

Coating a cationic antibacterial layer on the surface of cotton fabric is an effective strategy to provide it with excellent antibacterial properties and to protect humans from bacterial cross-infection. However, washing with anionic detergent will inactivate the cationic antibacterial coating. Although this problem can be solved by increasing the amount of cationic antibacterial coating, excessive cationic antibacterial coating reduces the drapability of cotton fabric and affects the comfort of wearing it. In this study, a coordinated antibacterial coating strategy based on quaternary ammonium salt and a halogenated amine compound was designed. The results show that the antibacterial effect of the modified cotton fabric was significantly improved. In addition, after mechanically washing the fabric 50 times in the presence of anionic detergent, the antibacterial effect against *Staphylococcus aureus* and *Escherichia coli* was still more than 95%. Furthermore, the softness of the obtained cotton fabric showed little change compared with the untreated cotton fabric. This easy-to-implement and cost-effective approach, combined with the cationic contact and the release effect of antibacterial agents, can endow cotton textiles with durable antibacterial properties and excellent wearability.

## 1. Introduction

Breathable and comfortable cotton fabric is one of the most popular choices for clothing worn in daily life [1,2]. Cotton benefits from its a high absorption ability and can easily absorb sweat, metabolites and sebum from the sweat/sebaceous glands of the skin. However, these secretions may provide a favorable environment for the growth of microorganisms such as bacteria and fungi [3]; therefore, these microorganisms can proliferate rapidly under certain conditions, and may pose a threat to public health.

In order to effectively control the microorganisms and reduce possible bacterial infections, the introduction of antibacterial materials is an effective strategy to eliminate bacteria and avoid serious infections [4]. In recent years, a variety of antibacterial agents such as chitosan [5], metal oxides [6], quaternary ammonium salts [7], peptides [8], and guanidine polymers [9] have been used in antibacterial finishing for cotton fabrics. According to the literature [10,11], cationic polymers such as quaternary ammonium salts exhibit excellent bactericidal performance, for example, cotton fabrics treated with quaternary ammonium salt macromolecules can directly kill bacteria by destroying the integrity of cell membranes and impairing the normal respiratory function of bacterial cells [12,13]. However, the cationic antibacterial agents can be inactivated when anionic polymers or additives are encountered [14].

As a disinfectant, N-haloamine compounds have many unique advantages, such as stability in a wide temperature and humidity range, durability in long-term use, and reproducibility after bleaching treatment [15]. More importantly, they do not affect the antibacterial effect when anionic compounds are encountered. Because the amide, imide and guanidine functional groups on the L-arginine molecule have a significant antibacterial effect after halogenation, in this work, L-arginine was chosen as the precursor of N-haloamine antibacterial molecules. L-arginine coating is able to maintain the original physical and mechanical properties of cotton fabric to the greatest extent, and has good biocompatibility [16], hence it does not cause irritation when it is in contact with human skin.

In order to consider the strength of the combination of the haloamine precursor and the matrix material and also its effect on the durability of the antibacterial effect of the material, the current work is divided into three main steps. L-arginine was modified by methacrylic anhydride (M-Arg), and then the cotton fabric was combined with modified arginine via covalent bonding. Finally, the M-Arg coated cotton fabric underwent a halogenation reaction. The results show that the cotton fabric obtained by this method had durable antibacterial activity after being washed 50 times in the presence of anionic detergent, and the antibacterial effect against both *Staphylococcus aureus* (*S. aureus*) and *Escherichia coli* (*E. coli*) was more than 95%. In addition, the treated cotton fabric can kill bacteria by direct contact and by destroying and releasing halogen ions to oxidize cell membranes. Besides, this contact/release coordinated antibacterial method does not affect the original properties of the cotton fabric.

## 2. Results

### 2.1. Synthesis of Cotton Fabrics Treated with CDDA and Its Physical Properties

Dimethyl dodecyl [3-(trimethoxysilyl) propyl] ammonium chloride (CDDA), a cationic organosilicon quaternary ammonium salt has been proved to be a practical antibacterial finishing agent [17]. CDDA was utilized to modify the surface of cotton fabrics in order to provide the fabric with durable antibacterial properties. Figure 1a shows that both the raw cotton fabric and cotton fabric modified with organosilicon antibacterial agent (2% cotton) have a smooth surface. As shown in Figure 1b, with the increase in the feed radio of the cationic organosilicon quaternary ammonium salt from 1% to 9%, the average bacteriostatic rate of the corresponding 1% cotton, 2% cotton, 3% cotton, 6% cotton, and 9% cotton fabric was 86.22%, 93.41%, 99.96%, 99.99%, 99.99% against *S. aureus*, and 82.12%, 88.78%, 92.12%, 99.65%, 99.99, 99.99% against *E. coli*, respectively. However, when the cotton fabric was washed with anionic detergent in water, the antibacterial function of organosilicon quaternary ammonium salt was inactivated to varying degrees. As presented in Figure 1b,c, the antibacterial property of 1% cotton, 2% cotton, 3% cotton, 6% cotton, 9% cotton fabric against *S. aureus* and *E. coli* was reduced to 42.21%, 48.63%, 72.35%, 89.96% and 96.56%, and 35.45%, 42.32%, 56.35%, 86.36%, 94.56%, respectively. As shown in Figure 2, the cotton fabric became stiffer and rougher with the increase in the amount of CDDA coating, and the water static contact angle of the modified cotton fabric increased from 98.6° to 132.7°, which significantly decreases the comfort of the cotton fabric. As a result, although the CDDA makes the cotton fabric durable and provides excellent antibacterial functions, the excessive organosilicon coating inevitably affects the original, good wearability of cotton fabric.

### 2.2. Preparation of N-Halamine-Containing Cotton Fabrics

Figure 3 shows images of the distribution of elements on the surface of the cotton fabrics after being washed 50 times with anionic detergent in water. It could be clearly seen that their morphologies did not change significantly after washing, and all the cotton fabrics samples still have a relatively smooth surface (Figure 3a). The elemental distribution of the modified cotton fabrics were detected by SEM and EDX (Figure 3b). The elements, including C, O, N, and Si can be seen on the surface of the haloaminated modified cotton fabric along the fiber, while the Cl elemental signal is scattered in the corresponding region. This is because chlorine ions can be released from cotton fabrics. The elemental signal of N has almost the same distribution as that of C and O, which indicates that there is almost no release of N.

To further explore the composition of the surface of cotton fabrics finished with antibacterial agents, Fourier transform infrared spectrometer (FTIR) was carried out. As shown in Figure 3c, the characteristic bands of CCDA at 2125 cm^−1^ (Si-H) and 769 cm^−1^ (Si-C) were observed from the curve for the coating of CCDA on the surface of the cotton fabric. After being modified with M-Arg, new peaks were found at 1640 cm^−1^, 1452 cm^−1^, and 1535 cm^−1^, which are attributable to C=O, C-N stretching and N-H bending vibration, respectively. For the bleached cotton fabric with sodium hypochlorite, a new peak of N-Cl (839 cm^−1^) appeared and the original N-H peak disappeared (Figure 3d). All of these results suggested that a coating based on cationic polymers and haloamide compounds was present on the surface of cotton fabrics.

### 2.3. Contact/Release Coordinated Antibacterial Properties of Cotton Fabrics Containing N-Halamine

Generally, the antibacterial pathways of cotton fabric based on the halogenation reaction can be classified as contact killing and release killing as illustrated in Figure 4a,b. To further check for the presence of the contact killing mechanism, bacterial cells were treated with N-halamine-containing cotton fabrics in the absence of liquid medium. The antibacterial results are displayed in Figure 4c and raw cotton fabrics were used as control. The survival rate of bacteria on the pure cotton fabrics was less than 70%. Unlike the raw cotton, the inhibition rate of the cotton-1 fabrics treated with CDDA, was 79.1% and 86.3% against *E. coli* and *S. aureus*, respectively, while the N-halamine-containing cotton fabrics (cotton-2) showed an inhibition rate of over 93.3% and 91.2% against *E. coli* and *S. aureus*, respectively. Due to the excellent antibacterial effect of haloamine compounds, by increasing the content of haloamide antibacterial coating, the antibacterial effect of N-halimane-containing cotton fabrics became even stronger. The inhibition rate of cotton-2, cotton-3, and cotton-4 was 93.3%, 98.9%, 99.9% against *S. aureus* and 91.2%, 97.6%, 99.9% against *E. coli*, respectively. An inhibition zone assay was carried out to further confirm the killing mechanism. As confirmed in previous reports, the antibacterial materials that utilize contact killing hardly show any inhibition zone [18]. As shown in Figure 4d, all of the N-halamine-containing cotton fabric samples show the inhibition area around the sample, while there was no inhibition zone on the raw cotton and cotton-1 fabrics (Figure S3).

Figure 5 shows the antibacterial performance of cotton fabrics after being washing 50 times with anionic detergent in water. In Figure 5a, it can be seen that less bacterial colonies grew on agar plates after treatment with antibacterial cotton fabric compared with raw cotton. After washing with anionic detergent in water, the inhibition rate of cotton-1, cotton-2, cotton-3 and cotton-4 was 55.41%, 89.22%, 95.6%, 99.962% against *E. coli* and 68.20%, 91.40%, 96.54%, 99.97% against *S. aureus*, respectively (Figure 5b).

### 2.4. Antibacterial Performance of Modified Cotton Fabrics after Washing with Anionic Detergent in Water

The live/dead bacterial fluorescence staining assay was also used to characterize the antibacterial properties. The bacteria were stained with a cell-permeant SYBR Green (SG) dye, which can stain the nucleic acids of both intact and permeabilized cells. The dead bacteria were counterstained with propidium iodide (PI) red dye, a cationic fluorescent dye. As shown in Figure 6a,b, numerous live *S. aureus* and *E. coli* were found to be green after being in contact with the raw cotton fabrics, whereas few bacteria were found in red. In contrast, after exposure to treated cotton fabrics (cotton-1, cotton-2 and cotton-3), the number of red dots were significantly increased, and all green color cells were almost exclusively dyed in red color, revealing the excellent antibacterial activity of cotton fabrics treated with antibacterial agent.

Field emission scanning electron microscopes (FESEM) were used to observe the change in the morphology of the bacteria. As exhibited in Figure 6c, bacterial cells of both *E. coli* and *S. aureus* cultured with raw cotton fabric were viable and had a smooth and integral cell wall structure. In contrast, the bacterial cells exposed to cotton-1 fabrics (finished with CDDA only) were partly deformed with a smooth surface. When the bacteria experienced N-Cl bonding on cotton fabrics containing N-halamine, both bacterial cells suffered from widespread cell lysis and a rough bacterial surface could be observed, which was caused by the strong oxidation of chloride ions. Figure 6d showed the redox reactions involved in (CH_3_)_2_N-Cl bonding, in this process the cotton fabrics containing N-halamine were first immersed into a water system and shaken over a week. The chlorine content in the water system was measured by iodometric/thiosulfate titration. The reaction and the corresponding color changes are shown in Figure 6d. The N-Cl first oxidizes iodide ions to produce iodine, and then the iodine is depleted by the reduction in the titrated thiosulfate and the color fades gradually.

It has been reported that the (CH_3_)_2_N-Cl can return to their precursor compounds when they are treated with bacteria in solution system [19,20], therefore the (CH_3_)_2_N-Cl was recovered after the simple halogenation. In order to examine the characteristics of the (CH_3_)_2_N-Cl, a recycle antibacterial test was performed using cotton-3 fabrics. After completion of the antibacterial test, the cotton-3 fabrics samples were collected and immersed in water for 5 days and then immersed in chlorinated cotton-3 fabrics with sodium hypochlorite solution (100 mL, 2 wt %) for 20 min. The antibacterial activities of the chlorinated samples were also evaluated using the plate counting method. After 10 cycles, the reduction in both *E. coli* and *S. aureus* remained as high as 96% after treatment with cotton-3 fabrics (as shown in Figure 7a). Moreover, no significant difference was observed in the bending length and bending stiffness of the cotton-3 fabrics before and after each cycle (Figure 7b,c). Compared to the pure cotton fabric (bending length 3.9 cm and bending stiffness 1.6 mN·cm), the softness of the cotton-3 fabric did not decrease much, which suggested that the wearability was good via this strategy.

## 3. Discussion

Due to their excellent wearability, which includes qualities such as air and moisture permeability, softness, warmth and good biocompatibility, cotton fabrics are one of the most commonly used fabrics in the apparel, decorative and industrial fields [13,21]. To further improve the added value of cotton fabrics, many research groups have devoted themselves to creating antibacterial finishing for cotton fabrics [22,23,24]. Among the antibacterial finishing agents, quaternary ammonium salt cationic polymer is a common antibacterial agent [25,26,27]. Mao et al., synthesized ester-containing cationic silicone softeners and coated it on cotton fabric, and found that the cotton fabric obtained good antibacterial activity against both gram-negative and gram-positive bacteria [28]. Liu et al., found that the antibacterial and hydrophobic properties of cotton fabrics treated with polysiloxane quaternary ammonium salt were enhanced [29]. Quaternary ammonium salt polymers are now easily available to use on cotton fabrics to establish complete killing bacteria sequences; however, knowledge regarding their antibacterial properties after washing with anionic detergents is fairly limited. In our study, dimethyl dodecyl [3-(trimethoxysilyl) propyl] ammonium chloride (CDDA) was chosen as the quaternary ammonium salt antibacterial agent and was coated on the surface of cotton fabrics in order to study the antibacterial effect of cotton fabrics after they were washed with anionic detergents in water.

CCDA has excellent stability, surface activity, emulsification, sterilization, disinfection, softness and antistatic properties [30]. By testing the antibacterial performance of cotton fabrics modified with CCDA, we found that the cationic antibacterial coating endowed the cotton fabric with a durable antibacterial effect; this is because the CCDA can coated on cotton fabric by covalent bonding [31,32]. Furthermore, even after washing 50 times in anionic detergent water, it had little impact on the softness of the cotton fabric coated with CCDA. Even when the washing cycles of the cotton fabric were increased up to 100 times, the bending stiffness of 1% cotton, 2% cotton, 3% cotton, 6% cotton, and 9% cotton was only reduced from 1.60, 2.3, 2.6, 5.7 mN·cm before washing to 1.73, 2.23, 2.53, 4.2, 5.01 mN·cm, respectively, (as shown in Figure S4), which indicates there is strong bond between the fabric and the CCDA agent. However, after washing with anionic detergent, all of the cotton fabrics coated with CDDA antibacterial agent lost their good antibacterial effect (Figure 1). Although increasing the content of the cationic antibacterial agents coating on the surface of cotton fabric helped to prevent the gradual loss of antibacterial activity after washing with anionic detergent, excessive cationic coating can affect the wearing comfort of the cotton fabric itself. In Figure 2, it can be seen that when the cationic antibacterial agent content increases, the hydrophilicity and softness of the cotton fabric decreases.

The N-haloamides characterized so far have exhibited the advantages of fast sterilization, high sterilization efficiency, storage stability, and reproducible antibacterial effects. As reported earlier, when the halogen amine compound is loaded onto fabric, it is able to acquire efficient sterilization effects [33]. Our study has further proved that N-haloamide can also have an antibacterial effect when it is grafted onto cotton fabrics.

In order to solve the problem of the inactivation of the antibacterial function in the cationic antibacterial agent when it encounters anionic detergent, N-halamine and cationic antibacterial agent were coated on cotton fabric to design a coating for a contact/release coordinated antibacterial pathway. Firstly, cotton fabrics were treated with cerium ammonium nitrate as an initiator in water, then, cationic antibacterial agent CDDA and arginine monomer with unsaturated carbon–carbon double bonding (M-Arg) were added (Figures S1 and S2). Treating cotton fabric with cerium ammonium nitrate can introduce free radicals onto the surface. After heating in water, the M-Arg and CCDA were grafted onto the surface of cotton fabric by free radical polymerization and polycondensation, respectively. As shown in Figure 3, a smooth coating was formed on the surface of the cotton fabric by heating and amide bond functional groups on the coating surface were halogenated, thus completing the preparation of the contact/release coordinated antibacterial cotton fabric. Cationic antibacterial agents can cause an uneven charge on the bacterial cell membrane, leading to cell cracking, and cytoplasmic leakage to kill bacteria [34]. N-haloamide can produce Cl^+^ ions to kill bacteria by direct contact with bacteria [35]. The existence of N-halamine and the cationic antibacterial agent not only adsorbs bacteria in close contact with the haloamine compound, but also takes advantage of the contact/release coordinated antibacterial action to effectively kill bacteria. More importantly, it resolves the issue of the failure of the antibacterial effect in fabrics finished with cationic antibacterial agent after washing in anionic detergent. As shown in Figure 5, all of the cotton fabrics exhibited excellent antibacterial effects. For example, the antibacterial rate after anion washing showed the highest rate of 99.9% against both *S. aureus* and *E. coli*. However, cationic antibacterial agents such as chitosan or quaternary ammonium salts can only exert antibacterial effects through a contact antibacterial pathway, and their antibacterial effects are greatly reduced when they encounter anionic polymers. Both metal oxides and N-halamine can continuously release antibacterial ions to kill bacteria, but the ability of metal oxides to kill bacteria does not last while the antibacterial effect of haloamide compounds can be recovered after simple halogenation.

To explain the mechanism of the cotton fabrics based on halogenation reaction, freeze-dried bacterial cells were treated with N-halamine-containing cotton fabrics to test for contact killing bacteria [33]. According to the reports in the literature [35,36], due to the negative charge of the bacterial cell membrane, the cationic antibacterial coating can have close contact with bacteria to kill them (as shown in Figure 4a). As shown in Figure 4b, unlike the cationic antibacterial action, the main antibacterial mechanism of the haloamides is the release of strong oxidizing chloride ions that act on the bacteria membrane [37,38,39]. However, through our contact antibacterial experiment, we found that the antibacterial effect of N-halamine-containing cotton fabrics was greater than that of the cotton fabric treated only with cationic antibacterial agent (CDDA) (Figure 4c,d); this shows that when the antibacterial coating was in close contact with bacteria, the (CH_3_)_2_N-Cl chemical bonding on the surface of the cotton fabric also releases strong oxidizing chloride ions to kill bacteria. Moreover, by EDX analysis, it was also found that the Cl element on the surface of the N-halamine-containing fabric was scattered in the corresponding region, while the C, O and N elemental signals were kept their original fiber-shaped appearance, which might be attributable to the release of chlorine ions from the cotton fabric (Figure 3). That all the N-halamine-containing fabrics displayed an obvious zone of inhibition was also important evidence for the release of killing bacteria. In Table S1, it can be seen that the Cl^+^ ion content reduced gradually reduced with the increase in the washing times. After washing 50 times, the Cl^+^ ion content on 0.5 g of cotton fabric dropped to below 0.1%, although the antibacterial effect of cotton fabrics can still reach above 90% against both *S. aureus* and *E. coli*. When the washing times were increased up to 100, all of the cotton fabrics’ antibacterial effect decreased to below 85% (shown in Figure S5), which suggests that if the washing times continue to increase, cotton fabric modified with antibacterial agents may not maintain excellent antibacterial properties as in the case of repeat washing in anionic detergent water. However, according to the GB/T 20944.3-2008 standard, the antibacterial activity of N-halamine-containing fabrics after 50 washes met the requirements of antibacterial textiles. Because there is no Cl^+^ release from cotton fabrics treated with CCDA (Table S2), their antibacterial effect is not significant after washing with anionic detergent in water (Figure 1). Moreover, compared with untreated cotton fabric, cotton fabrics coated with CCDA and haloamide compounds still had good softness even after 50 washes with anionic detergent (shown in Figure S6). Microscopy to detect live and dead bacteria confirmed that even after washing with anionic detergent, the cotton fabric still had high-efficiency antibacterial abilities. By analyzing the bacterial morphology of the cotton fabric after antibacterial treatment, we found that N-halamine-containing cotton fabrics not only destroyed the integrity of the bacterial cell membrane but also act by oxidizing on the surface of bacterial cells membrane. In addition, after bleaching with sodium hypochlorite, the antibacterial effects of the cotton fabric can be recycled, and the softness of the fabric does not change much after treatment, thus, cotton fabric treated with this strategy effectively solves the problem of the failure of the antibacterial function in the cationic antibacterial coating washed with cationic detergent.

## 4. Materials and Method

### 4.1. Material

L-Arginine, methacrylic anhydride and dimethyl dodecyl [3-(trimethoxysilyl) propyl] ammonium chloride (CDDA) were purchased from Aladdin Industrial Inc (No.809 Chuhua Branch Road, Fengxian, Shanghai 201417, China). Cerium ammonium nitrate [Ce(NH_4_)_2_(NO)_3_], 10% sodium hypochlorite solution (NaClO), sodium bicarbonate, and absolute alcohol were obtained from Tianjin Chemical Reagent Plant (Tianjin, China). All the chemicals were used without purification. *Escherichia coli* (*E. coli* ATCC 8099) and *Staphylococcus aureus* (*S. aureus* ATCC 6538) were purchased from Nanjing Clinical Biological Technology Co., Ltd. (Nanjing, China). 100% cotton fabric (wrap density: 228 ends cm^−1^, weft density: 165 picks cm^−1^, fabric 0.25 mm, areal density: 245 g m^−2^) was provided by Xiajin Renhe Textile Technology Co., Ltd. (Dezhou, China).

### 4.2. Synthesis of Modified L-Arginine with Carbon–Carbon Double Bond (M-Arg)

According to the relevant literature [40], L-arginine (8.7 g, 0.05 mol) and sodium bicarbonate (8.4 g, 0.1 mol) were added into a 250 mL two-necked flask containing 100 mL distilled water. Then, methacrylic anhydride (18.5 g, 0.12 mol) was added dropwise. The solution was stirred for 2 h in an ice bath and the pH of solution was adjusted to 7.4 with aqueous ammonia. Finally, the solution was extracted three times with dichloromethane. The white powders were produced after freeze-drying at −50 °C in vacuum. The yield was 62.1%.

### 4.3. Preparation of Antibacterial Cotton Fabric with Dimethyl Dodecyl [3-(T Rimethoxy-Silyl) Propyl] Ammonium Chloride

The different feed ratio of the cationic antibacterial agent, dimethyl dodecyl [3-(trimethoxysilyl) propyl] ammonium chloride was added into 20 mL water to prepare the solutions with concentrations of 1%, 2%, 3%, 6%, 9%. Then the cotton fabric samples (10 cm × 10 cm, 10 g) were added into cationic antibacterial agent solution and left for 8 h. After reaction, cotton fabrics were washed with deionized water and dried at 80 °C. Finally, the antibacterial 1% cotton, 2% cotton, 3% cotton, 6% cotton, and 9% cotton fabric samples were prepared, corresponding to 1%, 2%, 3%, 6%, 9% concentrations of cationic antibacterial agent.

### 4.4. Preparation of Antibacterial Cotton Fabrics Based on M-Arg Halogenation Reaction

For the synthesis of M-Arg grafted cotton fabric, cotton fabric samples (10 cm × 10 cm) were immersed in 200 mL aqueous solution and 0.5 g cerium nitrate was added. The mixture reacted at 60 °C for 30 min in an N_2_ atmosphere, the cotton fabric was taken out and washed three times with fresh deionized water, then the cotton fabrics were transferred into 250 mL aqueous solution, and M-Arg and dimethyl dodecyl [3-(trimethoxysilyl) propyl] ammonium chloride (DDA) were added, and kept for 12 h at the 70 °C in an N_2_ atmosphere. After the cotton fabric was dried at 60 °C, the cotton fabrics were immersed in 100 mL sodium hypochlorite solution for 10 min. The finally antibacterial cotton fabric samples were obtained after washing and drying. The preparation parameters are shown in Table 1.

The SEM image of the synthesized NPs was characterized by a JEM-2100F. X-ray Photoelectron Spectroscopy (XPS) measurements were carried out with a commercial spectrometer (Thermo, ESCALAB 250). The stiffness of the cotton fabric was tested by a LFY-207 automatic fabric stiffness tester (40 × 250 mm, 3–5 mm/s).

### 4.5. Antibacterial Activity Assessment

#### 4.5.1. Contact Killing Assay

The freeze-dried bacterial cells of *E. coli* and *S. aureus* were collected by centrifugation [33], washed twice with pure water and then freeze-dried under vacuum for 24 h to a dry powder. The dried bacteria were cultured for 12 h at 37 °C in a dry aseptic environment and then placed on the surface of the cotton fabric samples. After having contact for 24 h, the bacterial powder was washed off the cotton fabrics and suspended in 10 mL of fresh LB nutrient broth. Finally, the survival of bacteria was determined using the plate counting method.

#### 4.5.2. Determining the Inhibition Rate of Antibacterial Fabrics

The colony count method was used to determine the antibacterial activity of cotton fabric samples, in accordance with ISO20743-2007, bacteria (*S. aureus*, *E. coli*) were grown overnight at 37 °C under agitation (200 rpm) in Luria-Bertani (LB) growth medium. Pure PBS as the control sample and cotton fabrics (0.75 g) treated with antibacterial agent were cut into pieces and added to a shaking bed to culture at 37 °C for 24 h, and then 500 μL of culture medium was taken out and serially diluted to give a very dilute culture of bacteria, which was plated onto solidified LB agar plates and incubated at 37 °C for 24 h. After 24 h, the number of bacterial colonies on the plates was counted and the inhibition rate was evaluated by the following Equation (1).

(1) $$Y=\frac{W_{t}-Q_{t}}{W_{t}}\times 100\%$$

where *W_t_* is the number of bacterial colonies in the control sample; and *Q_t_* is the number of colonies of cells treated with antibacterial cotton fabrics.

### 4.6. Bacteria Cells Morphology Observation with SEM

The bacteria (*S. aureus*, *E. coli*) were cultivated in the LB broth overnight in an oven at 37 °C and then the activated bacteria in the LB broth (10 mL) were centrifuged at 5000 rpm for 10 min in a centrifuge tube and the supernatant was removed by washing with PBS. Then 40 mL of PBS and 0.5 g of cotton fabric were added into this centrifuge tube, and shaken for 4 h (130 r/min, 37 °C). Finally, phosphate buffer (pH 7.4; 10 mL) containing 2.5% glutaraldehyde was added to the centrifuge tubes and then placed in the fridge overnight at 4 °C to fix the bacterial morphology. A drop of bacterial solution taken from the tubes on a silicon wafer was left to dry completely at room temperature and then coated with gold by sputtering for a SEM observation.

### 4.7. Confocal Laser Scanning Microscopy (CLSM) for Detection of Live/Dead Bacteria

Different antibacterial cotton fabric samples were added into a 10 mL bacteria solution (10^8^ CFU/mL) and then centrifuged at 5000 rpm for 15 min, the supernatant was removed and PI and SG DNA dye were added at a concentration of 10 μg/mL. After staining for 20 min, the bacteria were washed two times with PBS buffer. Then, the suspension was spotted on a microscope slide and examined using a laser scanning confocal microscope (LeicaDMI8).

### 4.8. The Test of Cl^+^ Ion Content on N-Halamine-Containing Cotton Fabrics

The cotton fabric (0.5 g) was cut into pieces and put into 20 mL deionized water solution, then potassium iodide (0.5 g) and starch solution (2 mL, 1 wt %) were added and stirred at room temperature for 30 min. Finally, sodium thiosulfate solution (0.001 mol/L) was used to titrate. After the solution was colorless, the amount of sodium thiosulfate was recorded and the following formula was used to calculate the active chlorine content of the sample. Each sample was titrated three times. The calculation formula for the active chlorine (Cl^+^) content in the sample is as follows:

(2) $$Cl^{+}(\%)=\frac{Ν\times V\times 35.45}{W\times 2}$$

where *N* is the equivalent concentration of sodium thiosulfate solution for titration (mol/L); *V* is the volume of sodium thiosulfate solution consumed (mL); and *W* is the weight of the sample (g).

## 5. Conclusions

In this study, we first prepared a layer of cationic antibacterial coating on the surface of cotton fabric using a common silicone quaternary antibacterial agent. The antibacterial performance of the cotton fabric gradually decreased after washing with anionic antibacterial agent. Increasing the content of cationic antibacterial coating helped to prevent the problem of antibacterial activity failure, but the cotton fabric felt stiff and rough and would not be comfortable to wear. Based on this, a synergistic antibacterial strategy based on cationic contact and a halogenated antibacterial agent releasing method for the construction of antibacterial coatings on cotton fabrics was designed. The antibacterial effect of cotton fabrics treated by this method is significant and it has no obvious effect on the softness of the fabric. More importantly, after 50 mechanical washes with anionic detergents, the antibacterial properties of the modified cotton fabrics against *Staphylococcus aureus* and *Escherichia coli* still reached more than 96%, which is an important reference value in the field of functional modification of textiles.

## Figures and Tables

**Figure 1:** (**a**) The optical and SEM images of raw cotton fabrics and cotton fabrics finished with CDDA. The bar is 10 µm. (**b**) The antibacterial properties of cotton fabrics against *S. aureus* (**c**) and *E. coli* after washing 50 times with the addition of anionic detergent. Q-cotton fabrics were washed with pure water, N-cotton fabrics were washed with anionic detergent in water.

**Figure 2:** The water contact angle and bending rigidity of cotton fabric modified with cationic antibacterial agent.

**Figure 3:** (**a**) The SEM photograph of cotton fabric samples. (**b**) Mapping results of the elements on the surface of cotton-4 fabric washed with anionic detergent. (**c**) FTIR spectra of cotton fabrics before haloamination reaction, A: untreated cotton fabric, B: cotton fabric finished with dimethyl dodecyl [3-(trimethoxysilyl) propyl] ammonium chloride (CDDA), C–E: cotton fabric modified with CCDA and L-Arginine containing carbon–carbon double bond (M-Arg). (**d**) FTIR spectra of cotton fabric modified with CCDA and M-Arg after haloamination reaction.

**Figure 4:** The antibacterial mechanism of contact killing (**a**) and release killing (**b**) for antibacterial cotton fabrics. (**c**) Quantitative analysis of antibacterial properties of cotton fabrics after washing them 50 times without adding anionic detergent. (**d**) The inhibition zones of antibacterial cotton fabrics, the bar is 2 cm.

**Figure 5:** The antibacterial performance of cotton fabrics after being washed 50 times with anionic detergent in water. Cotton-1 fabric was treated with only dimethyl dodecyl [3-(trimethoxysilyl) propyl] ammonium chloride (CDDA); cotton-2, cotton-3 and cotton-4 fabric samples were the N-halamine containing antibacterial fabrics. (**a**) Photographs of the bacterial colony growing on an agar plate. (**b**) The inhibition rate of different cotton fabric samples.

**Figure 6:** (**a**) The assessment of live/dead *S. aureus* (**a**) and *E. coli* (**b**) treated with different cotton fabrics. The bar is 20 µm, green dots represent alive and dead *S. aureus* or *E. coli*; the red dots represent dead *S. aureus* or *E. coli*. (**c**) The SEM images of bacterial cell morphology exposed to different cotton samples. (**d**) Oxidation-reduction reactions and the corresponding color change involved in the iodometric/thiosulfate titration.

**Figure 7:** (**a**) Antibacterial activity of cotton-3 fabrics against *E. coli* and *S. aureus* during five antibacterial cycles. Bending length (**b**) and bending stiffness (**c**) in the softness test of cotton-3 fabrics.

**Table 1:** The parameters for the preparation of antibacterial cotton fabric samples.

Name Code	M-Arg (g)	DDA (g)	Cotton Fabrics (g)	NaClO (mL)	H_2_O (mL)
Cotton-1		0.1	10	20	250
Cotton-2	0.1	0.1	10	20	250
Cotton-3	0.2	0.1	10	20	250
Cotton-4	0.3	0.1	10	20	250

## Supplementary Materials

The supplementary materials are available online at https://www.mdpi.com/1422-0067/21/18/6531/s1.
